The article "Antibiofilm Synergistic Activity of Streptomycin in Combination with Thymol-Loaded Poly (Lactic-co-glycolic Acid) Nanoparticles against Klebsiella pneumoniae Isolates" was published in 2022. Journal: Evid Based Complement Alternat Med.

# Antibiofilm Synergistic Activity of Streptomycin in Combination with Thymol-Loaded Poly (Lactic-co-glycolic Acid) Nanoparticles against *Klebsiella pneumoniae* Isolates

**DOI:** 10.1155/2022/1936165

**Published:** 2022-07-21

**Authors:** Borel Ndezo Bisso, Christian Ramsès Tokam Kuaté, Nathalie Boulens, Eric Allémann, Florence Delie, Jean Paul Dzoyem

**Affiliations:** ^1^Department of Biochemistry, Faculty of Science, University of Dschang, Dschang, Cameroon; ^2^School of Pharmaceutical Sciences, University of Geneva, Geneva, Switzerland

## Abstract

**Background:**

Thymol is an important component of essential oils found in the oil of thyme, is extracted mainly from *Thymus vulgaris*, and was shown to act synergistically with streptomycin against *Klebsiella pneumoniae* biofilms. Additionally, thymol could be encapsulated into poly (lactic-co-glycolic acid) (PLGA) nanoparticles to overcome issues related to its low water solubility and high volatility. The present study aimed to investigate the antibiofilm activity of thymol-loaded PLGA nanoparticles (Thy-NPs) alone and in combination with streptomycin against biofilms of *K. pneumoniae* isolates.

**Methods:**

The broth microdilution method was used to determine the minimum inhibitory concentration (MIC) and minimum bactericidal concentration (MBC). The antibiofilm activities were determined by the safranin dye assay. The synergistic effect of Thy-NPs with streptomycin was assessed by the checkerboard method. The kinetic study of the biofilm biomass and time-kill assay were further performed.

**Results:**

Thy-NPs exhibited the highest antibacterial activity against *K. pneumoniae* isolates, with MIC values ranging from 1 to 8 *µ*g/mL. Additionally, Thy-NPs showed the highest antibiofilm activity against *K. pneumoniae* isolates with minimal biofilm inhibitory concentration (MBIC) and minimal biofilm eradication concentration (MBEC) values ranging from 16 to 64 *µ*g/mL and from 32 to 128 *µ*g/Ml, respectively. The combination treatment combining Thy-NPs with streptomycin showed a synergistic effect against the inhibition of biofilm formation and eradication of biofilms of *K. pneumoniae* isolates with fractional inhibitory concentration index values ranging from 0.13 to 0.28. In addition, the MBIC and MBEC values of streptomycin against *K. pneumoniae* isolates were dramatically reduced (up to 128-fold) in combination with Thy-NPs, suggesting that Thy-NPs would enhance the antibiofilm activity of streptomycin. The biomass and time-kill kinetics analysis confirmed the observed synergistic interactions and showed the bactericidal activity of streptomycin in combination with Thy-NPs.

**Conclusions:**

Our results indicate that the synergistic bactericidal effect between streptomycin and Thy-NPs could be a promising approach in the control of biofilm-associated infections caused by *K. pneumoniae*.

The article "Antibiofilm Synergistic Activity of Streptomycin in Combination with Thymol-Loaded Poly (Lactic-co-glycolic Acid) Nanoparticles against Klebsiella pneumoniae Isolates" was published in 2022. Journal: Evid Based Complement Alternat Med.

## 1. Introduction

*Klebsiella pneumoniae* is a Gram-negative, encapsulated, nonmotile, rod-shaped pathogenic bacterium, and member of the Enterobacteriaceae family that can cause various types of healthcare-associated infections, including bloodstream infections, pneumonia, meningitis, wound or surgical site infections, and urinary tract infections. *Klebsiella* bacteria are normally found in the human intestines (where they do not cause disease) and are also found in human feces [1]. *K. pneumoniae* is second to *Escherichia coli* the most important opportunistic human pathogen responsible for a wide spectrum of nosocomial and community-acquired infections [2]. *K. pneumoniae* can form biofilms, which are communities of bacteria that adhere to biotic or abiotic surfaces and are encased in an extracellular matrix composed of polysaccharides, proteins, and extracellular DNA that protect the bacteria from harsh environmental conditions. The biofilm lifestyle provides more resistance to antibiotics (10–1000 times more resistant than planktonic form) and the host immune system than their planktonic counterparts [3]. Biofilm formation is one of the major causes of infection persistence particularly in medical device-related infections. The resistance of biofilms to antibiotics may be associated with limited diffusion of antibiotics through the biofilm matrix, the transmission of resistance genes, the lower growth rate of bacteria, the overexpression of efflux pumps, and persistent cells in biofilms [4, 5]. Combination therapies and exploring natural compounds are good strategies to overcome this problem.

Thymol is the principal monoterpene phenol occurring in essential oils isolated from plants belonging to the Lamiaceae family (*Thymus*, *Ocimum,* and *Origanum*). Previous studies have shown that thymol presents several pharmacological properties such as antioxidant, antiviral, antifungal, antibacterial, and antibiofilm [6]. Thymol interacts with the lipidic bacterial membrane via direct binding with the biomolecules providing strong antimicrobial activity by disrupting the localization of membrane-associated proteins and the permeability of the bacterial cell membranes. Additionally, thymol reduces the biomass of biofilms, prevents adhesion, and destroys the structure of biofilms by modulating the quorum sensing system [6, 7]. Thymol was reported to reduce the amount of biofilm of *Pseudomonas aeruginosa* within the range of 70–77% and 52–75% for *Staphylococcus aureus* [8]. In another study, thymol significantly inhibited 88% of methicillin-resistant *Staphylococcus aureus* (MRSA) biofilm formation at 100 *μ*g/mL, reduced the surface adherence of MRSA, and enhanced the antibacterial and biofilm eradication efficiency of rifampicin against MRSA [9]. In addition, our recent studies reported a synergistic antibiofilm effect between thymol and aminoglycosides against *K. pneumoniae* and *Salmonella enterica* biofilms [10, 11]. The association of thymol with antibiotics showed a strong synergistic effect both in the inhibition of biofilm formation and the destruction of the preformed biofilm of *K. pneumoniae*, with the minimum biofilm inhibitory concentration (MBIC) and the minimum biofilm eradication concentration (MBEC) values of streptomycin being reduced by 16- to 64-fold [10].

The article "Antibiofilm Synergistic Activity of Streptomycin in Combination with Thymol-Loaded Poly (Lactic-co-glycolic Acid) Nanoparticles against Klebsiella pneumoniae Isolates" was published in 2022. Journal: Evid Based Complement Alternat Med.

Despite the excellent therapeutic potential of thymol, its clinical application is still limited due to its low solubility and high volatility. The low solubility of a bioactive substance decreases its bioavailability. Bioactive substances with poor bioavailability are not unable to reach the minimum effective concentration to exhibit therapeutic action [12]. Many nanoparticles for antimicrobial drug delivery have been widely explored over the last few decades. In particular, poly (lactic-co-glycolic acid) (PLGA) nanoparticles have various advantages (biocompatibility and biodegradability) in the nanotechnology field. Its ability to enhance drug pharmacokinetics and bioavailability, by protecting the drug against inactivation by enzymes, by targeting and penetrating cell membranes and biofilms, or by favoring a sustained drug release while limiting side effects, makes this system considered a promising strategy for overcoming biofilm-associated infections [13, 14]. It was demonstrated that PLGA nanoparticles containing xylitol successfully penetrated the extracellular polymeric substance (EPS) matrix, promoting antibiofilm activity due to their unique physicochemical properties and enhanced penetration in biofilm EPS [15]. In addition, the combination of nanoparticle-encapsulated bioactive molecules deriving from plants with antibiotics may lead to effective synergy against antibiotic resistance [16]. The synergistic effects of nanoparticles associated with antibiotics may increase antimicrobial efficiency to combat multidrug-resistant microbes via several mechanisms, including membrane disruption, and binding to cellular machinery essential for transcription and protein synthesis [17].

In our previous study, we demonstrated that thymol could act synergistically with streptomycin to inhibit the biofilm formation and eradicate the preformed biofilm of *K. pneumoniae* [10]. We also showed that thymol could be encapsulated into PLGA nanoparticles to overcome issues related to its low water solubility and high volatility [18]. Therefore, we hypothesized that Thy-NPs may be used to substantially improve the antibiofilm properties of streptomycin, allowing its use for the effective treatment of *K. pneumoniae* biofilm infections. Thus, the present study was undertaken to investigate the antibacterial and antibiofilm potential of thymol-loaded poly (lactic-co-glycolic acid) nanoparticles alone, and in combination with streptomycin against *K. pneumoniae* biofilms. We also investigated the mechanism of this synergistic effect by analyzing the kinetics of the biofilm biomass as well as the time-kill kinetics of the viable cells.

The article "Antibiofilm Synergistic Activity of Streptomycin in Combination with Thymol-Loaded Poly (Lactic-co-glycolic Acid) Nanoparticles against Klebsiella pneumoniae Isolates" was published in 2022. Journal: Evid Based Complement Alternat Med.

## 2. Materials and Methods

### 2.1. Chemicals, Reagents, and Nanoparticles

The following chemicals were purchased from Sigma Aldrich: streptomycin, thymol with a purity of ≥98.5, dimethyl sulfoxide (DMSO), and p-iodonitrotetrazolium chloride (INT). PLGA (lactide: glycolide 50 : 50, Mw 24000–38000, Resomer RG 503H) was purchased from Boehringer Ingelheim Pharma GmbH&Co. The following culture media were acquired from Dominique Dutscher: Mueller Hinton Agar (MHA) and Mueller Hinton Broth (MHB).

The thymol-loaded PLGA nanoparticles (Thy-NPs) used in this work were prepared, and their physicochemical properties were determined in our previous study [18]. Therefore, the thymol loading capacity obtained was considered in the Thy-NPs concentrations used in all the assays.

### 2.2. Bacteria

Clinical isolates of *K. pneumoniae* from urine samples, namely, *Kp02*, *Kp03*, *Kp04*, *Kp05,* and *Kp55* were used in the present study and provided by Pr. Fotsing Pierre from the Laboratory of Microbiology (“*Université des Montagnes*,” Cameroon). One strain of *K. pneumoniae* (ATCC 13882) used in the present study was obtained from the American Type Culture Collection.

### 2.3. Determination of the Minimal Inhibitory Concentration (MIC) and Minimal Bactericidal Concentration (MBC)

The antimicrobial activity of Thy-NPs against planktonic *K. pneumoniae* was assessed using the broth microdilution method [19, 20]. Stock solutions of Thy-NPs and streptomycin were prepared by dissolving each compound in distilled water to final concentrations of 4096 *μ*g/mL and 1024 *µ*g/mL for Thy-NPs and streptomycin, respectively. Serial dilutions (1 : 2) of stock solution were made from 2048 to 1 *μ*g/mL for Thy-NPs and 512 to 0.125 *μ*g/mL for streptomycin using MHB at a total volume of 100 *µ*L per well in a 96-well microplate. Then, 100 *µ*L of bacterial inoculum (1.5 × 10^6^ CFU/mL) was added to each well and the microplate was incubated at 37°C for 24 hours. The final concentrations of Thy-NPs and streptomycin ranged from 1024 to 0.5 *µ*g/mL and 256 to 0.125 *µ*g/mL, respectively. After incubation, 40 *µ*L of INT solution (0.2 mg/mL) was added and the microplate was incubated at 37°C for 30 min. The positive control contained broth mixed with bacterial inoculum, while the blank control contained broth only. The lowest concentration of Thy-NPs at which no color change occurred (yellow to pink color) was recorded as the MIC.

The article "Antibiofilm Synergistic Activity of Streptomycin in Combination with Thymol-Loaded Poly (Lactic-co-glycolic Acid) Nanoparticles against Klebsiella pneumoniae Isolates" was published in 2022. Journal: Evid Based Complement Alternat Med.

For the MBC test, an aliquot of 50 *µ*L from the wells that showed no bacterial growth was added to a microplate containing 150 *µ*L of MHB, and then the microplate was incubated for 48 h at 37°C. The MBC was considered as the lowest concentration of Thy-NPs that showed no color change after the addition of INT, as mentioned above. The experiment was carried out in triplicate and repeated three times.

### 2.4. Biofilm Formation Assay

Based on the kinetic metabolic activity of biofilm formation in a previous study [10], the biofilm biomass of *K. pneumoniae* isolates was determined with a colorimetric method based on safranin dye [21]. Briefly, 100 *µ*L of bacterial inoculum (1.5 × 10^6^ CFU/mL) and 100 *µ*L of MHB supplemented with 2% glucose were added to a 96-well flat-bottomed polystyrene plate. After incubation for 24 h at 37°C, the plate was washed three times with phosphate-buffered saline (PBS, pH 7.2) to remove the planktonic cells, and biofilms were fixed with methanol for 20 min at room temperature. After incubation, the methanol was removed and the biofilm was stained with 150 *µ*L of safranin (1%). After incubation for 15 min at room temperature, the excess safranin was removed, and the dye bound to the adherent cells was solubilized with 150 *µ*L of 95% ethanol. Wells containing MHB supplemented with 2% glucose were used as negative controls. To quantify biofilm biomass, the optical density (OD) was measured at 570 nm using a microplate reader (SpectraMax 190, Molecular Devices). The intensity of biofilm formation was classified as follows: non-biofilm producer (OD ≤ ODc), weak biofilm producer (ODc < OD ≤ 2 × ODc), moderate biofilm producer (2 ODc < OD ≤ 4 ODc), and strong biofilm producer (4 × ODc < OD), where ODc is the optical density of the cut-off value, which is defined as the sum of the arithmetic mean of the negative control and threefold standard deviation.

### 2.5. Biofilm Inhibition Assay

The efficacy of Thy-NPs to inhibit biofilm formation was determined using the microtiter plate method as described by Teanpaisan et al. [22]. Stock solutions of Thy-NPs and streptomycin were prepared as described above. Serial dilutions (1 : 2) of stock solution were made from 2048 to 1 *μ*g/mL for Thy-NPs and 512 to 0.125 *μ*g/mL for streptomycin using MHB at a total volume of 100 *µ*L per well in a 96-well microplate. Then, 100 *µ*L of bacterial inoculum (1.5 × 10^6^ CFU/mL) was added to each well, and the microplate was incubated at 37°C for 24 h. The final concentrations ranged from 1024 to 0.5 *µ*g/mL and 256 to 0.125 for Thy-NPs and streptomycin, respectively. After incubation, the non-adherent cells were removed by washing the wells three times with PBS, and adherent cells were fixed with methanol for 20 min at room temperature. Then, the plates were treated for the biofilm formation assay as described above. The optical density was measured at 570 nm using a microplate reader. Untreated wells and wells containing broth only were used as positive and blank controls, respectively. The percentage inhibition of biofilm formation was calculated using the following equation: %inhibition = 100 − [(OD_test_ − OD_blank_)/(OD_control_ − OD_blank_) *×* 100]. The lowest concentration of Thy-NPs that reduces the biofilm biomass by 100% was considered as the minimal biofilm inhibitory concentration (MBIC). The test was performed three times in triplicate.

The article "Antibiofilm Synergistic Activity of Streptomycin in Combination with Thymol-Loaded Poly (Lactic-co-glycolic Acid) Nanoparticles against Klebsiella pneumoniae Isolates" was published in 2022. Journal: Evid Based Complement Alternat Med.

### 2.6. Biofilm Eradication Assay

The efficacy of Thy-NPs against preformed biofilms was performed based on a previous protocol [21]. Stock solutions of Thy-NPs and streptomycin were prepared as described above. Then, biofilms were formed for 48 h at 37°C using the biofilm formation method as described above. After washing with PBS, serial twofold dilutions of 200 *µ*L of Thy-NPs or streptomycin (at concentrations ranging from 1024 to 0.5 *µ*g/mL and 256 to 0.125 *µ*g/mL, respectively) were added to the wells and the plate was incubated for 24 h at 37°C. After incubation, the plate was treated as described above and the minimal biofilm eradication concentration (MBEC) was defined as the lowest concentration of Thy-NPs that completely eradicate (100%) the preformed biofilm.

### 2.7. Combination of Thy-NPs with Streptomycin against Biofilm Formation

The combined effects of Thy-NPs and streptomycin on inhibiting biofilm formation were evaluated by the checkerboard dilution method as described by Hu et al. with slight modifications [23]. Stock solutions of Thy-NPs and streptomycin were prepared by dissolving each compound in distilled water to final concentrations of 256 *µ*g/mL and 64 *μ*g/mL for Thy-NPs and streptomycin, respectively. First, 50 *µ*L of MHB supplemented with 2% glucose was added to a 96-well flat-bottomed polystyrene plate. Then, 50 *µ*L of Thy-NPs from the twofold serial dilution was added in the vertical row and 50 *µ*L of streptomycin from the twofold serial dilution was added in the horizontal row. To each well, 100 *µ*L of bacterial inoculum (1.5 × 10^6^ CFU/mL) was added and the plate was incubated at 37°C for 24 h. The Thy-NPs and streptomycin concentrations used ranged from 32 to 0.5 *µ*g/mL and 8 to 0.0078125 *µ*g/mL, respectively. After incubation, the plate was washed three times with PBS and treated as described above. The MBIC of each compound in combination was determined and the fractional inhibitory concentration index (FICI) was calculated as follows: FICI = (MBIC of streptomycin in combination/MBIC of streptomycin alone) + (MBIC of Thy-NPs in combination/MBIC of Thy-NPs alone). The FICI results were interpreted as follows: synergy (FICI ≤0.5), additivity (0.5 < FICI ≤1), indifference (1 < FICI ≤ 4), and antagonism (FICI > 4) [23]. Fold reduction in MBIC of streptomycin was calculated as follows: Fold reduction = MBIC of streptomycin/MBIC of streptomycin + Thy-NPs.

The article "Antibiofilm Synergistic Activity of Streptomycin in Combination with Thymol-Loaded Poly (Lactic-co-glycolic Acid) Nanoparticles against Klebsiella pneumoniae Isolates" was published in 2022. Journal: Evid Based Complement Alternat Med.

### 2.8. Combination of Thy-NPs with Streptomycin against Preformed Biofilm

The interaction of Thy-NPs and streptomycin against preformed biofilms was also determined by the checkerboard dilution method as described by Hu et al. with some modifications [23]. Biofilms were formed in a 96-well flat-bottomed polystyrene plate for 48 h as described above, and then the plate was washed thrice with PBS to remove non-adherent cells. The plate was then filled with 100 *µ*L of MHB supplemented with 2% glucose and treated with each compound as described above. The MBEC, FICI, and fold reduction in MBEC of streptomycin were determined as described above.

### 2.9. Kinetic Analysis of the Biofilm Biomass and Time-Kill Assay

The rate of the prevention of biofilm biomass formation and the dispersion rate of the mature biofilm biomass by the combination of thy-NPs with streptomycin were monitored according to a previously described method with slight modifications [24]. For the kinetics of the inhibition of biofilm formation, after treatment and incubation at different time points (3, 6, 9, 12, 18, and 24 h at 37°C), the medium was discarded and the plate was washed three times with PBS. Then, the plates were treated as described above. Wells with MHB only and untreated wells containing bacteria were served as the blank and positive controls, respectively. For the kinetic of the destruction of mature biofilm, after biofilm formation for 48 h as described above, the planktonic cells were removed by washing thrice with PBS. Then, the plate was treated with Thy-NPs and streptomycin alone or in combination. After incubation for different time points (1, 2, 3, 4, 5, and 24 h at 37°C), the plate was treated as described above.

The article "Antibiofilm Synergistic Activity of Streptomycin in Combination with Thymol-Loaded Poly (Lactic-co-glycolic Acid) Nanoparticles against Klebsiella pneumoniae Isolates" was published in 2022. Journal: Evid Based Complement Alternat Med.

To confirm the synergistic antibiofilm activities of Thy-NPs and streptomycin, a time-kill kinetic study was performed by estimating the surviving cells in the biofilm using the viable plate count method [25]. After different points of treatment, the medium was discarded and the plate was washed three times with PBS. Then, the adherent cells were suspended in PBS by scraping, followed by serial dilution and 100 *µ*L of each dilution sample was plated on the MHA plate. After incubation of the MHA plate at 37°C for 48 h, the bacterial colonies were counted and results were expressed as log10 CFU/mL. A bactericidal effect was defined as ≥3 log10 reduction in the colony count compared with the positive control. Synergy was defined as ≥2 log decrease in CFU/mL at 24 h by combination treatment in comparison with their single agent [24].

### 2.10. Statistical Analysis

Each experiment was performed in triplicate and the results are shown as means ± standard deviation (SD). To determine statistically significant differences, a one-way analysis of variance (ANOVA) was performed using GraphPad Prism software version 8.0. The *p* value < 0.05 was considered statistically significant.

## 3. Results

The nanoparticles were prepared using a single-emulsion solvent evaporation method. The nanoparticle size was approximatively 190 nm with a polydispersity between 0.069 and 0.104 and zeta potential ranging from −1.2 to −9.5 mV [18].

### 3.1. Antimicrobial Activity of  Thy-NPs  against Planktonic Cells of *K. pneumoniae*

The MIC and MBC of Thy-NPs were assessed against the five *K. pneumoniae* isolates, and the data are shown in Table 1. The MIC and MBC values obtained against planktonic cells ranged from 1 to 8 *µ*g/mL and 4 to 32 *µ*g/mL, respectively. As shown by their respective ratios, the MIC and MBC values of Thy-NPs were 32- to 64-fold and 8- to 128-fold decreased, respectively, when compared with free thymol. Empty PLGA nanoparticles did not affect bacterial growth (MIC and MBC >1024 *µ*g/mL).

### 3.2. Biofilm Biomass Production

The OD values obtained from the quantitative analysis of biofilm biomass production are shown in Figure 1. Based on ODc = 0.38 all the *K. pneumoniae* isolates were able to form biofilms. The *Kp02* (OD = 1.59 ± 0.08) and *Kp04* (OD = 1.64 ± 0.081) isolates were classified as strong biofilm producers, while the *Kp03* (OD = 1.29 ± 0.06), *Kp05* (OD = 1.14 ± 0.04), and *Kp55* (OD = 1.2 ± 0.02) isolates were classified as moderate biofilm producers. However, the *K. pneumoniae* ATCC 13882 strain was classified as a weak biofilm producer. Strong and moderate biofilm-producing isolates of *K. pneumoniae* were selected for antibiofilm assays.

The article "Antibiofilm Synergistic Activity of Streptomycin in Combination with Thymol-Loaded Poly (Lactic-co-glycolic Acid) Nanoparticles against Klebsiella pneumoniae Isolates" was published in 2022. Journal: Evid Based Complement Alternat Med.

### 3.3. Antibiofilm Effect of Thy-NPs Alone and in Combination with Streptomycin

#### 3.3.1. Inhibition of Biofilm Formation (Prevention of Initial Bacterial Cell Attachment)

Thy-NPs inhibited bacterial cell attachment with MBIC values ranging from 16 to 64 *µ*g/mL. In our previous study, MBIC values of free thymol ranged from 256 to 1024 *μ*g/mL [10]. The MBIC values of Thy-NPs were 8 to 64 times lower than those of free thymol that were obtained in our previous study. The MBIC values varied from 4 to 8 *μ*g/mL for streptomycin. When Thy-NPs were combined with streptomycin against biofilm formation, synergy was observed in all five isolates tested, with FICI values ranging from 0.13 to 0.28 with 32- to 128-fold reduction in the MBIC values of streptomycin. The fold reduction in MBIC of streptomycin obtained with thymol encapsulated into nanoparticles was 2- to 3-fold higher than the fold reduction (16- to 64-fold) obtained with free thymol (Table 2).

#### 3.3.2. Disruption of Preformed Biofilm (Destruction of Mature Biofilm Mass)

Thy-NPs dispersed the mature biofilm of *K. pneumoniae* isolates with MBEC values ranging from 32 to 128 *µ*g/mL. The MBEC values of Thy-NPs were found to be 8 to 16 times lower than the free thymol (512 to 1024 *μ*g/mL), which was obtained in our previous study. MBEC values varied from 32 to 128 *μ*g/mL for streptomycin. The combination of Thy-NPs and streptomycin also induced a synergistic effect (FICI = 0.13–0.28) against all isolates of *K. pneumoniae* with a 32- to 128-fold reduction in MBEC values of streptomycin. The fold reduction in MBEC of streptomycin combined with Thy-NPs was increased two times compared with free thymol (16- to 64-fold) (Table 3).

### 3.4. Kinetic Analysis of the Biofilm and Time-Kill Assay

#### 3.4.1. Kinetic and Time-Kill Assay of the Biofilm Formation

Figure 2 shows the kinetic results of biofilm biomass formation by *K. pneumoniae* treated with Thy-NPs and streptomycin alone and in combination. It was observed that the combination of Thy-NPs and streptomycin effectively suppressed (*p* < 0.05) the biofilm formation of all isolates of *K. pneumoniae* from time zero compared with Thy-NPs or streptomycin alone and the control group. When used separately at the same concentration as in the synergy, Thy-NPs and streptomycin showed an increase in biofilm biomass formation over time, with optical density values up to 0.8 at 24 hours.

Similar results were obtained by CFU count in the time-kill study (Figure 3). The use of streptomycin alone displayed no reduction in CFU count. However, the combination of Thy-NPs and streptomycin induced significant (*p* < 0.05) cell death with ≥2 log10 reduction from 3 hours to ≥3 log10 reduction after 18 hours against all the isolates.

The article "Antibiofilm Synergistic Activity of Streptomycin in Combination with Thymol-Loaded Poly (Lactic-co-glycolic Acid) Nanoparticles against Klebsiella pneumoniae Isolates" was published in 2022. Journal: Evid Based Complement Alternat Med.

#### 3.4.2. Kinetic and Time-Kill Assay of the Biofilm Destruction

The kinetic of biofilm destruction revealed that over 24 hours, the combination of Thy-NPs and streptomycin significantly destroyed (*p* < 0.05) the biomass of the mature biofilm of all isolates of *K. pneumoniae* compared to Thy-NPs or streptomycin alone (Figure 4). The breakup of the biomass started after 2 hours for *Kp03* and after 1 hour for all other isolates when treated with nanoparticles alone or in combination with streptomycin. After 3–4 hours, the biofilm biomass was completely dispersed by the combination with OD values of zero, while the OD value of Thy-NPs alone remained between 0.7 and 1.2.

The time-kill study of *K. pneumoniae* during biofilm destruction over 24 hours showed a similar trend to the kinetics of biomass destruction (Figure 5). Thy-NPs alone displayed greater activity against the killing of viable cells in mature biofilm biomass than streptomycin alone. Thy-NPs alone or in combination with streptomycin showed a decrease in the number of cells counts biofilm. The killing of *K. pneumoniae* cells in the biofilm started at the first hour, and the number of CFU/mL remained approximately 4 log10 over 24 hours in the treatment with Thy-NPs alone, while this number dropped to an undetectable level in the treatment with a combination after 3 to 4 hours.

## 4. Discussion

Biofilm-related infections caused by *K. pneumoniae* are recalcitrant and associated with limited treatment options. Therefore, it is important to develop new therapeutic strategies to prevent biofilm formation or eliminate mature biofilms [4]. Thymol is the major component found in the essential oils from *Thymus vulgaris*, and other plants such as *Ocimum gratissimum* and *Carum copticum* [6]. It has attracted much attention owing to its ability to prevent biofilm formation or eliminate mature biofilms [8, 9]. In addition, thymol has also displayed synergistic activities with streptomycin against *K. pneumoniae* biofilms [10]. In this study, thymol was encapsulated into PLGA nanoparticles to increase its antibacterial and antibiofilm properties, and then it was combined with streptomycin as a starting point for developing new therapeutic strategies against biofilm-associated infections. First, we investigated the antibacterial effect of Thy-NPs against planktonic cells of *K. pneumoniae.* It was observed that the MIC and MBC values for thymol-loaded PLGA nanoparticles were significantly lower than those obtained with free thymol. These results indicated that the Thy-NPs formulations had an increased antibacterial effect compared with free thymol. The increased antibacterial activity of Thy-NPs compared with free thymol could be due to the reduced Thy-NPs size (190 nm). The particle size of Thy-NPs could increase their penetration inside the cell membrane of bacteria, resulting in more damage in the cell [14]. In addition, the phenolic hydroxy group of thymol enhanced its hydrophilic property, leading to inhibition of bacterial growth and even killing them [6]. Improved efficacy of drug-loaded PLGA nanoparticles and intracellular delivery of drugs on different microbial strains have been reported by several studies. For instance, PLGA nanoparticles loaded with curcumin showed greater antibacterial activity on different bacterial strains than free curcumin [26]. Additionally, Lacoma et al. reported significant antimicrobial activity of cloxacillin-loaded PLGA nanoparticles compared to free cloxacillin against *Staphylococcus aureus* [27]. Cardamom oil-loaded chitosan nanoparticles were found to exhibit excellent antimicrobial potential against extended-spectrum lactamase-producing *Escherichia coli* and methicillin-resistant *Staphylococcus* aureus [28]. However, empty PLGA nanoparticles had no antimicrobial activity on bacterial growth.

The article "Antibiofilm Synergistic Activity of Streptomycin in Combination with Thymol-Loaded Poly (Lactic-co-glycolic Acid) Nanoparticles against Klebsiella pneumoniae Isolates" was published in 2022. Journal: Evid Based Complement Alternat Med.

Although *K. pneumoniae* is well-known for its ability to form biofilms, this ability was also assessed for our isolates. The results showed that *K. pneumoniae* isolates were strong and moderate biofilm producers. The different levels of biofilm production in *K. pneumoniae* isolates could be explained by the different expression levels of genes involved in the different steps of biofilm formation [29].

The antibiofilm activity of Thy-NPs against *K. pneumoniae* isolates was investigated. Thy-NPS showed better potential to prevent biofilm formation and eliminate mature biofilms of *K. pneumoniae* isolates than free thymol. The higher antibiofilm activity of Thy-NPs may be due to the size and surface charge of nanoparticles. The nanoparticle size substantially impacts the diffusion of Thy-NPs into the biofilm matrix, leading to more damage to the biofilm cells. The nanoparticle's surface charge can be responsible for specific biofilm targeting by electrostatic interactions with the biofilm matrix, favoring the attachment of nanoparticles to the biofilm matrix and resulting in the release of the drug inside the biofilm [15, 30]. Additionally, the nanoparticle's high surface-area-to-volume ratio could enable high penetration of the drug, which may result in stronger antibiofilm efficacy [31]. These results corroborate those obtained by Klodzińska et al. and Iannitelli et al. [32, 33]. However, there was no difference in the imbibition of biofilm formation or eradication of biofilm between the control (no treatment) and PLGA (empty) control, indicating that empty PLGA nanoparticles had no antibiofilm activity. The MBEC values of Thy-NPs were higher than their MBIC values. These results could be due to the presence of persistent cells with slow or absent growth within biofilms that are also not destroyed by Thy-NPs treatment [34]. Another contributing factor may be the overexpression of the efflux pump by sessile biofilm-forming cells [35].

The article "Antibiofilm Synergistic Activity of Streptomycin in Combination with Thymol-Loaded Poly (Lactic-co-glycolic Acid) Nanoparticles against Klebsiella pneumoniae Isolates" was published in 2022. Journal: Evid Based Complement Alternat Med.

Our study also revealed a synergistic effect of Thy-NPs and streptomycin against biofilm formation and mature Biofilms in all *K. pneumoniae* isolates tested. In addition, the concentration of streptomycin was significantly decreased and its antibacterial activity was significantly increased when combined with Thy-NPs compared to streptomycin alone. The synergistic effect obtained may be due to the inhibition of quorum sensing or dispersion of biofilms by Thy-NPs, increasing bacterial susceptibility to streptomycin. Data on synergistic effects of antibiotics and natural products loaded into biodegradable and biocompatible nanoparticles such as PLGA are very scarce. However, several studies have reported synergistic interactions between antibiotics and nanomaterials [36, 37].

To confirm the synergistic antibiofilm activity of Thy-NPs in combination with streptomycin, and assess the bactericidal mode of action, kinetic and time-kill assays of biofilm formation and disruption were performed. The Thy-NPs combined with streptomycin showed a synergistic effect with bactericidal activity, illustrated by a remarkable reduction in the cell count over time, both in biofilm biomass formation and in biofilm biomass destruction for all isolates of *K. pneumoniae* tested. The synergistic activity of Thy-NPs and streptomycin is a strong advantage, as current strategies are often inefficient to kill or restrict the growth of the cells in the biofilm. However, neither Thy-NPs nor streptomycin alone exhibited bactericidal activity against *K. pneumoniae* biofilms.

Our findings described above suggested that the synergistic effect of Thy-NPs and streptomycin is achieved both by inhibiting the initial attachment of *K. pneumoniae* for the formation of biofilms and by the destruction of the extracellular polymeric matrix, thus increasing the susceptibility of suspended *K. pneumoniae* cells to streptomycin. The use of Thy-NPs combined with streptomycin can be a promising strategy to combat antibiotic resistance and biofilms of *K. pneumoniae*.

## 5. Conclusion

This study demonstrated for the first time the antibacterial and antibiofilm effects of thymol nanoparticles against *K. pneumoniae*. Moreover, the combination of encapsulated thymol with streptomycin enhanced the synergistic effect against *K. pneumoniae* biofilms. Additionally, our results indicate that the synergistic bactericidal effect could be a promising approach in the control of biofilm-associated infections caused by *K. pneumoniae*. Taken together, our results indicate that streptomycin combined with Thy-NPs could be further developed as an antibiofilm agent.

The article "Antibiofilm Synergistic Activity of Streptomycin in Combination with Thymol-Loaded Poly (Lactic-co-glycolic Acid) Nanoparticles against Klebsiella pneumoniae Isolates" was published in 2022. Journal: Evid Based Complement Alternat Med.

## Figures and Tables

**Figure 1:** Biofilm biomass of *K. pneumoniae* isolates. Isolates were divided into two groups based on the cut-off value of OD_C_: strong biofilm producer (SBP), moderate biofilm producer (MBP), and weak biofilm producer (WBP). The dashed line represents the value of optical density of control (OD_C_) at 570 nm.

**Figure 2:** Kinetic of *K. pneumoniae* isolates biofilm biomass formation in the presence of Thy-NPs and streptomycin alone and in combination. Thy-NPs: thymol-laded PLGA nanoparticles; Strep: streptomycin. Data represent the average values and standard deviation of three independent experiments.^*∗*^Significant difference between the combination and single drug (*p* < 0.05).

**Figure 3:** Time-kill kinetic study of Thy-NPs and streptomycin alone and in combination against *K. pneumoniae* isolates biofilm biomass formation. Thy-NPs: thymol-loaded nanoparticles; Strep: streptomycin. Data represent the average values and standard deviation of three independent experiments.^*∗*^Significant difference between the combination and the single drug (*p* < 0.05).

**Figure 4:** Kinetic of *K. pneumoniae* isolates biofilm biomass destruction in the presence of Thy-NPs and streptomycin alone and in combination. Thy-NPs: thymol-loaded PLGA nanoparticles; Strep: streptomycin. Data represent the average values and standard deviation of three independent experiments.^*∗*^Significant difference between the combination and the single drug (*p* < 0.05).

**Figure 5:** Time-kill kinetic study of Thy-NPs and streptomycin alone and in combination against *K. pneumoniae* isolates biofilm biomass destruction. Thy-NPs: thymol-loaded PLGA nanoparticles; Strep: streptomycin. Data represent the average values and standard deviation of three independent experiments.^*∗*^Significant difference between the combination and the single drug (*p* < 0.05).

**Table 1:** MIC and MBC (*µ*g/mL) of Thy-NPs and free thymol against planktonic cells of *K. pneumoniae.*

Isolates	Thymol^*∗*^		Thy-NPs				Empty NPs	
	MIC	MBC	MIC	MBC	R1	R2	MIC	MBC
*Kp02*	128	256	4	16	32	16	>1024	>1024
*Kp03*	64	512	1	4	64	128	>1024	>1024
*Kp04*	128	256	8	32	16	8	>1024	>1024
*Kp05*	256	512	8	16	32	32	>1024	>1024
*Kp55*	128	512	2	8	16	64	>1024	>1024

MIC: minimum inhibitory concentration, MBC: minimum bactericidal concentration, ^*∗*^data from the previous study [10], Thy-NPs: thymol loaded-PLGA nanoparticles, Empty NPs: empty PLGA nanoparticles, R1: MIC of Thy-NPs/MIC of free thymol, and R2: MBC of Thy-NPs/MBC of free thymol.

The article "Antibiofilm Synergistic Activity of Streptomycin in Combination with Thymol-Loaded Poly (Lactic-co-glycolic Acid) Nanoparticles against Klebsiella pneumoniae Isolates" was published in 2022. Journal: Evid Based Complement Alternat Med.

**Table 2:** MBIC and FICI of combined Thy-NPs with streptomycin against inhibition of biofilm formation of *K. pneumoniae*.

Isolates	MBIC (*µ*g/mL)			FICI/Int	Fold reduction	
	Alone		Combined			
	Strep^#^	Thy-NPs	Strep + Thy-NPs		Strep	Thy-NPs
*Kp02*	4	32	0. 125 + 8	0.28/S	32-fold	4-fold
*Kp03*	4	16	0.0625 + 2	0.14/S	64-fold	8-fold
*Kp04*	4	64	0.125 + 8	0.16/S	32-fold	8-fold
*Kp05*	8	32	0.0625 + 4	0.13/S	128-fold	4-fold
*Kp55*	8	16	0.0625 + 4	0.26/S	128-fold	4-fold

MBIC: minimal biofilm inhibitory concentration, FICI: fractional inhibitory concentration index, Int: interpretation, Strep: streptomycin, Thy-NPs: thymol-loaded PLGA nanoparticles, Strep^#^: data from the previous study [10], and S: synergy.

**Table 3:** MBEC and FICI combined Thy-NPs with streptomycin against the eradication of biofilm of *K. pneumoniae*.

Isolates	MBEC (*µ*g/mL)			FICI/Int	Fold reduction	
	Alone		Combined			
	Strep^#^	Thy-NPs	Strep + Thy-NPs		Strep	Thy-NPs
*Kp02*	32	128	0.25 + 16	0.13/S	128-fold	8-fold
*Kp03*	64	32	2 + 8	0.28/S	32-fold	4-fold
*Kp04*	64	64	1 + 16	0.27/S	64-fold	4-fold
*Kp05*	128	64	2 + 8	0.14/S	64-fold	8-fold
*Kp55*	32	128	0.25 + 16	0.13/S	128-fold	8-fold

MBEC: minimal biofilm eradication concentration, FICI: fractional inhibitory concentration index, Int: interpretation, Strep: streptomycin, Thy-NPs: thymol loaded-PLGA nanoparticles, Strep^#^: data from the previous study [10], and S: synergy.

## Data Availability

The data used to support the findings of this study are available upon reasonable request to the corresponding author.
